# Application of a Nursing Data-Driven Model for Continuous Improvement of PICC Care Quality

This article has been retracted.

**DOI:** 10.1155/2022/7982261

**Published:** 2022-03-19

**Authors:** Juzhen Zhou, Lihua Wang

**Affiliations:** ^1^Department of Oncology,Dushu Lake Hospital, Soochow University, Suzhou 215000, Jiangsu, China; ^2^Department of Oncology, The First Affiliated Hospital of Soochow University, Suzhou 215000, Jiangsu, China

## Abstract

A PICC catheter maintenance network was established and managed to monitor the maintenance of catheters in placed patients throughout the process, providing homogeneous PICC catheter continuity of care for patients. Model-driven thinking is an idea for simulation system development. Model-driven architecture (MDA) is a design methodology that implements model-driven thinking and is widely used in simulation system development. Based on the requirements of nursing, the data-driven model is mainly divided into interface layer and functional service layer; this study adopts MDA technology which can detach the functions of the system from the platform, based on domain knowledge, and the metamodel adopts XSD-based data model to generate the PIM model, which is stored in the model library. The results showed that the number of nurses at maintenance sites increased from 79 to 232, the PICC placement rate for oncology patients increased from 35.0% to 76.0%, the nurse maintenance operation pass rate increased from 53.9% to 88.4%, and the maintenance default rate decreased from 40.0% to 10.9%.

## 1. Introduction

Peripherally inserted central catheters (PICC) are catheters placed via peripheral venous puncture into the superior or inferior vena cava at the tip. PICCs are widely used in clinical practice because they can avoid repeated punctures, reduce patient pain, reduce the occurrence of mechanical phlebitis, reduce the impact of chemotherapeutic drug extravasation on peripheral vessels, are simple and safe to operate, and provide intravenous access to oncology patients for medium-to long-term chemotherapy [1]. Catheter maintenance needs to be performed locally, and if timely and correct PICC maintenance cannot be achieved during discharge, it will cause complications such as blockage, phlebitis, and infection and prolong the PICC retention time, resulting in an increased rate of unplanned extubation [1].

PICC catheters have important application value for patients who need to receive long-term treatment such as intravenous injection, which can effectively reduce the number of venipuncture of patients, thus appropriately reducing the pain caused by frequent punctures and to a certain extent reducing the workload of nursing staff [2], which has high feasibility and efficiency in clinical care. However, in the actual application, patients are prone to various accidents during intubation, resulting in adverse events and complications, which have a serious impact on their therapeutic effects and physical and mental health. Therefore, continuous quality improvement of care during PICC placement is necessary and has a positive clinical effect on the effectiveness and safety of clinical treatment [3].

PICC not only effectively avoids direct contact between drugs and arm veins but also has become an important way of clinical treatment and parenteral nutrition because of its simple operation, easy maintenance, and long retention time [4]. However, in practice, improper care is likely to lead to the occurrence of accidents such as catheter blockage and dressing dislodgement, resulting in complications such as prolonged retention time and mechanical phlebitis, which seriously affects the clinical treatment of patients [5]. In this study, we applied the management method of intravenous therapy care team to the continuous quality improvement of PICC care, and the results showed that the observation group had a significantly higher rate of successful primary puncture and a significantly shorter retention time and lower complication rate than the control group. This shows that the intravenous therapy nursing team has significant application effect in continuous improvement of PICC nursing quality and is worth promoting [6].

As a typical nursing information application system, the development of simulation software for nursing data-driven model faces many problems such as uncertain requirements and rapid changes in the application environment [7], and new software development ideas and methods need to be explored. At present, the range constructs multiple sets of nursing data-driven models, which are applied to different simulation implementation platforms, such as RT-Space platform and DWK platform [8], resulting in serious waste of resources and increasing many repetitive tasks, and the main reason for this phenomenon is because the system does not have portability and reusability [9].

Therefore, in order to ensure the effectiveness and safety of PICC treatment, this study applies the intravenous therapy care team to the continuous improvement of PICC care quality and discusses the effect of its application.

## 2. Knowledge Background

### 2.1. PICC Catheter Maintenance Behavior

After the placement of PICC catheters, catheter maintenance can take several to dozens of times and weeks [10], and the safety and standardization of catheter maintenance is related to the length of catheter retention. Many patients need to travel long distances to return to our hospital for catheter maintenance after catheter placement, so it is especially important to establish a PICC maintenance site for patients nearby.

The regional collaborative care model of PICC maintenance, which was found during the preliminary piloting process, is a phased establishment of an integrated urban-rural PICC maintenance network, which, on the one hand, facilitates maintenance in the vicinity of patients (the return maintenance rate decreased from 71.9% in 2014 to 29.2% in 2017), and on the other hand, reduces catheter maintenance costs, reduces discomfort caused by long-distance travel, alleviates patient pain, and protects patient safety. For medical workers, it can realize the rational division of nursing work, improve work efficiency, enhance operational skills, decrease the rate of missing PICC maintenance (*P* < 0.01), increase the rate of qualified PICC maintenance, increase team cohesion, and improve nursing quality; for hospitals, it can reduce the incidence of nursing disputes, improve the rate of PICC placement, improve patient satisfaction, and enhance the overall brand image of hospitals; for society [11], it can reduce the incidence of nursing disputes, improve the rate of PICC placement, and improve the overall brand image of hospitals. For the hospital, it can reduce nursing disputes, improve PICC placement rate, improve patient satisfaction, and enhance the overall brand image of the hospital; for the society, it can effectively build a medical regional collaboration network, provide a reference for subsequent medical regional collaboration, alleviate the problem of concentration and uneven distribution of medical resources today, and achieve a win-win situation for both economic and social benefits [12].

### 2.2. PICC Maintains Regional Collaborative Care Model

Facilitating catheter maintenance for patients between treatments PICC reduces the number of venipunctures, avoids PICC has been widely accepted and used by oncology chemotherapy patients because it reduces the number of venous punctures, avoids damage to blood vessels from extravasation of chemotherapy drugs, reduces patients' psychological stress, and provides a safe intravenous access for treatment [13]. And the maintenance of catheters is related to whether patients can safely complete their treatment. The use of online platforms such as WeChat can strengthen the connection between nurses and between nurses and patients and ensure the continuity of care [14]. Before the catheter is placed, the PICC maintenance network allows for quick and easy access to the location of each maintenance site and informs patients of the maintenance site near their place of residence; after the catheter is placed, patients can receive efficient and standardized homogeneous nursing services at the nearest maintenance site through the regional nursing collaboration model, saving patients' time and expenses such as travel and accommodation costs so that patients can enjoy “home” maintenance services. At the same time, patients can enjoy “doorstep” maintenance services, reduce their economic burden and psychological pressure, receive homogeneous services, reduce the risk of catheter-related complications, indirectly promote their physical recovery, and meet the needs of discharged patients for extended care services [15, 16], which is a safe and feasible nursing service model. This model improves patient satisfaction and win-win situation for both nurses and patients and promotes the development of the out-of-hospital care model [17].

### 2.3. PICC Maintains Regional Collaborative Care Model

The regional resource allocation was optimized by building a PICC maintenance network, leading from point to point, expanding the coverage of PICC maintenance to a certain extent, and breaking through the limitations of the original method; at the same time, through the development of relevant systems, the workflow of nurses at maintenance points was standardized, their knowledge of PICC was strengthened, the safety of nursing services was ensured, the qualification rate of catheter maintenance was improved, and the maintenance of catheters was improved. Quality prolongs the service life of PICCs, promotes the clinical application of PICC technology in oncology chemotherapy patients, and promotes the development of PICC specialist nurses [18]. In addition, the use of this nursing model has saved nurses' PICC maintenance time in tertiary hospitals, allowing nurses to have more energy to take care of inpatients, further improving inpatient satisfaction, enhancing the quality of departmental care and the overall image of hospitals, and also promoting the promotion of the graded diagnosis and treatment system.

## 3. Data-Driven Model Development Ideas

As a typical nursing information application system, the development and exploitation of its simulation software faces many problems such as uncertain requirements and rapid changes in the application environment [5], and new software development ideas and methods need to be explored. At present, the range constructs multiple sets of nursing data-driven models, which are applied to different simulation implementation platforms, such as RT-Space platform and DWK platform, resulting in serious waste of resources and increasing many repetitive tasks, and the main reason for this phenomenon is because the system does not have portability and reusability. The application of data model-driven development technology can realize the separation of application logic and underlying changes of the care data-driven model and increase the reuse of application logic and even application subsystems at large granularity, thus enhancing the adaptability and changeability of the software system and realizing that one modeling can be applied to different technical environments [7].

The requirements of the nursing data-driven model are mainly divided into the interface layer and the functional service layer. In this study, MDA technology can be used to detach the functions of the system from the platform, based on domain knowledge, and the metamodel is used to generate PIM models based on the XSD data model, which is deposited in the model library. The models proposed in the model library can all be mapped to different platforms, including RT-Space platform, DWK platform, HLA, and other specific platforms, and realize automatic code generation and rely on component technology to finally realize the development of the whole system; the main implementation framework is shown in Figure 1.

The combat system interface protocol-aided design tool was introduced in [6], which proposed a model-driven approach by converting the stored relevant combat system interface protocol unit data into an XML schema file (XSD). Therefore, the realization of a data model-centric simulation system development method in the MDA environment and the construction of a care data-driven model data model is a very important element.

## 4. Nursing Data-Driven Model

The nursing data-driven model is a very complex system, and the data model of the system plays a crucial role in the simulation development. During the development of the system using a model-driven approach, modifications to the data model can be automatically reflected in all phases of the design, such as updating system object properties, updating system interface protocols, updating the simulation model, and updating the implementation code of the simulation system.

### 4.1. XSD-Based System Data Model

In the development process of the nursing data-driven model, even though there is a better top-level design, the system design will still be adjusted as the user needs keep changing, the interface will keep changing, and the interface parsing needs to be adjusted significantly. The use of XML Schema definitions (XSD) to build the data model can solve the problem of adapting to such interface changes in the system development process, in order to improve the system development efficiency, reduce development costs, and make the interface with strong adaptability.

For the information units and related data fields defined in the nursing data-driven model interface protocol, the XSD is used to build a data model, which mainly describes the basic information of the model, the data types, and the component information of the model and describes the structural relationships between the information elements and the detailed information used to constrain each element, for example, the name, type, length, maximum value, and minimum value of the data fields. The information structure of the nursing data-driven model data model is shown in Figure 2.

#### 4.1.1. Model Basic Information

The basic information of the model describes the management class information such as the name of the nursing data-driven model simulation program model in English, the development language of the model, and the model development platform, and its information structure is shown in Figure 3.

#### 4.1.2. Model Component Information

Model component information describes model information such as model component description information, desired initialization parameters, attribute class input information, attribute class output information, event class input information, and event class output information of the care data drive model. The information structure is shown in Figure 4.

Among them, thought initialization information is used to describe the inherent properties of the simulation objects, such as the heading and speed of the target trajectory object of the care data-driven model. Attribute class information is used to describe the object class information of the interaction between simulation objects, such as the target trajectory information reported by radar. Event class information is used to describe the interaction class information between simulation objects, such as hard weapon target indication messages and radar status reporting messages [14].

### 4.2. Application of the Data Model in Interface Description

Combined with SOA thinking, the concept of service is introduced. A service can accept requests and send response results, and the format of the received request messages and the feedback response messages are defined from the XSD-based data model. When implementing a specific service, the distribution of that service over the network needs to be bound to a specific network communication protocol. The data model mainly describes the format and content of the messages in the interface, but it is necessary to add a description of the service interface information, i.e., a description of the operation, port, and protocol binding information.

## 5. A Data-Driven Model Approach to Nursing Data-Driven Model Development

Generally speaking, software code can be divided into three parts: generic code, personality code, and structural repetitive code. In the nursing data-driven model simulation software, the generic code is the basic code that contains the basic framework of the software and implements the simulation system; the personalized code is the code that implements the specific functions of the nursing data-driven model, and the structural repetitive code mainly contains the code that describes the specific format of the nursing data-driven model information messages and the message parsing procedure, and through further research, it is found that this part of the code is the structural repetitive code which contains code that describes the specific format of the nursing data-driven model messages and the message parsing procedure.

In the previous sections, the data model of the nursing data-driven model describes mainly the information related to messages. During the development process, there will be many structural repetitive codes in the nursing data-driven model, which can be generated by the conversion of the data model of the system. By establishing a mapping relationship between the data model and the structural repetitive codes and applying model-driven ideas to guide the automatic generation of this part of the code, the development efficiency of the nursing data-driven model can be greatly improved.

### 5.1. XSD-Based Message Parsing Code Generation

In order to realize the data-driven model code development, it is actually the realization of the conversion from PIM to actual code in MDA idea.

The XML file is defined in a tree-like structure, which is characterized by good structure and facilitates program analysis, and can be processed by tree traversal and generation algorithms. In order to improve the efficiency of the interface code development, the idea is based on the one shown in Figure 5. After reading the XSD file, the XSD file structure is first analyzed and the parsing code is generated according to the file structure.

### 5.2. PIM to PSM Conversion

The platform-independent model (PIM) is designed without considering the middleware platform on which the final implementation is made or the platform on which the final code will run; it is a model that describes the functions and structure of the system and does not include any platform technologies. The design of the platform-related model (PSM) is closely related to the specific platform, which depends on the functions and services provided by the platform and involves the implementation details of the system on the platform.

Examples of platforms include HLA, CORBA, and DWK, which are used in the simulation of the data-driven model of care. Converting PIM to PSM, that is, from a conceptual analytical model to a computer simulation, the implementation of the model can be automated by the PSM automatic conversion tool.

The conversion from a nursing data-driven model PIM to a PSM that satisfies the DWK platform implementation protocol requires the PIM to achieve the conversion to PSM in accordance with the object model structure, simulation drive method, service acquisition method, and exception mechanism and parameter type specified by DWK.

## 6. Case Study

### 6.1. PICC Maintenance Point Quality Control

The nursing department arranges for members of the sedation team to be assigned to the PICC maintenance sites in each region of Suzhou, forming one-to-one hospital commissioner-to-hospital contact, understanding the training needs of local nurses through PICC exchange groups, making training plan, and going to local hospitals to organize training every year. Every six months, the nursing department of the hospital takes the lead in conducting network theoretical and operational assessments for the nurses of PICC maintenance sites to ensure the correctness of nursing operations of the nurses at the maintenance sites and to ensure that the maintenance sites can provide quality services to patients. ① Network theory assessment: the theory assessment scores 100 points, 90 points, and makes up those who fail to pass the test. The system automatically closes after the time is up, and the test taker submits the test paper and the system automatically scores it to avoid the errors in the manual correction of the paper. Those who fail the examination have a chance to make up the 

### 6.2. Effectiveness of PICC Maintenance Network Implementation

According to the statistics of the Department of Medical Oncology of our hospital, the establishment of the regional PICC maintenance network has led to the increase in the number of PICC insertion year by year, and the triage of maintenance points has realized the maintenance of patients in the vicinity, which effectively reduces the rate of patients returning to the hospital for maintenance. The triage of maintenance points has enabled patients to be maintained close to each other and effectively reduced the rate of patients returning to the hospital for maintenance, as shown in Table 1.

The operation of nurses at maintenance sites in 2019 (the initial stage of PICC maintenance network construction) and 2020 (the middle stage of PICC maintenance network construction) was compared, and PICC maintenance videos were filmed by one to two nurses qualified in PICC maintenance at maintenance sites by means of online operation assessment. All participating nurses signed the informed consent form, and the operation videos were rated by our PICC specialist nurses, and the results showed that the operation level of nurses at the PICC maintenance site improved and the operation assessment pass rate increased (*P* < 0.01), see Table 2.

By comparing the rate of missing PICC maintenance with the rate of patient satisfaction, we surveyed patients who returned to the hospital for maintenance after PICC discharge in the medical oncology and radiotherapy departments, and the results showed that the rate of missing catheter maintenance decreased, various catheter-related complications decreased, and patient satisfaction increased year by year during the interval between treatments (Table 3).

Extended care service refers to the provision of nursing care and health guidance services for discharged patients with nursing needs, which is an extension of inpatient services [19]. The establishment of PICC maintenance network has solved the worries of discharged patients and provided patients with “home” care services. The “Health China 2030” plan outlines the establishment of information sharing and interconnection mechanisms, the continuous improvement of service networks, the improvement of the treatment-rehabilitation-long-term care service chain, and the standardization and promotion of “Internet + health care” services to realize the Health China Cloud Health Plan. The service plan is shown in Figure 6.

Although the establishment of PICC maintenance network based on regional nursing coordination has achieved the above results, there are still shortcomings; the regional distribution of PICC maintenance points has not yet fully covered all hospitals, especially some more remote areas. The effect of different PICCs is shown in Figure 7, and the future should strengthen the publicity, optimize the management of PICC maintenance network, gradually strengthen the maintenance team, while strengthening their own strength, and further expand the coverage of PICC maintenance network to further meet the needs of patients in rural areas. This model provides a reference for the subsequent implementation of graded diagnosis and treatment, incorporating more nursing content and medical models and realizing the sharing of medical and nursing resources.

## 7. Conclusions

The effectiveness of an intravenous therapy care team is continuously improving the quality of PICC care. A PICC catheter maintenance network was established and managed to monitor the maintenance of catheters in patients with catheters placed throughout the process, providing homogeneous PICC catheter continuity of care for patients. At the same time, PICC quality management standards are formulated for the actual situation, and the quality of placement is regularly supervised and evaluated; at the same time, the team is responsible for organizing training and assessment of relevant staff, conducting comprehensive discussions on difficult cases, proposing solutions, and conducting joint consultations when necessary.

## Figures and Tables

**Figure 1:** Block diagram of the simulation development of the nursing data-driven model.

**Figure 2:** Information structure of the nursing data-driven model.

**Figure 3:** Information structure of the basic information of the model.

**Figure 4:** Model component information structure.

**Figure 5:** Code generation parsing method.

**Figure 6:** PICC of different partition implementation effects.

**Figure 7:** Effectiveness of PICC care for different patient households.

**Table 1:** PICC placement rate and return maintenance rate in medical oncology department.

Particular year	Actual number of catheters	Catheterization		Maintain	
		Number of persons to be placed	Catheterization rate (%)	Number of returned maintenance personnel	Return to hospital maintenance rate (%)
2014	432	1235	35	311	71.9
2015	480	942	51	245	50.1
2016	521	766	68	188	63.1
2017	589	775	76	172	29.2

**Table 2:** PICC maintenance point and nurse maintenance operation assessment pass rate.

Particular year	Number of nurses	Qualified persons (person)	Pass rate (%)
2019	78	42	53.9
2020	232	205	88.4
*x* ^2^		42.948	
*P*		<0.001	

**Table 3:** PICC with tube patient maintenance absence rate and satisfaction survey.

Particular year	Number of patients examined	Maintenance missing		Satisfaction	
		Number of cases	Incidence (%)	Number of cases	Satisfaction rate (%)
2015	195	78	40	124	63.6
2016	238	26	10.9	229	96.3
*x* ^2^		49.651		79.756	
*P*		<0.001		<0.001	

## Data Availability

The data underlying the results presented in the study are available within the article.
